This article has been retracted.

# Suppression of uPAR Retards Radiation-Induced Invasion and Migration Mediated by Integrin β1/FAK Signaling in Medulloblastoma

**DOI:** 10.1371/journal.pone.0013006

**Published:** 2010-09-24

**Authors:** Arun Kumar Nalla, Swapna Asuthkar, Praveen Bhoopathi, Meena Gujrati, Dzung H. Dinh, Jasti S. Rao

**Affiliations:** 1 Department of Cancer Biology & Pharmacology, University of Illinois College of Medicine at Peoria, Peoria, Illinois, United States of America; 2 Department of Pathology, University of Illinois College of Medicine at Peoria, Peoria, Illinois, United States of America; 3 Department of Neurosurgery, University of Illinois College of Medicine at Peoria, Peoria, Illinois, United States of America; The University of Chicago, United States of America

## Abstract

**Background:**

Despite effective radiotherapy for the initial stages of cancer, several studies have reported the recurrence of various cancers, including medulloblastoma. Here, we attempt to capitalize on the radiation-induced aggressive behavior of medulloblastoma cells by comparing the extracellular protease activity and the expression pattern of molecules, known to be involved in cell adhesion, migration and invasion, between non-irradiated and irradiated cells.

**Methodology/Principal Findings:**

We identified an increase in invasion and migration of irradiated compared to non-irradiated medulloblastoma cells. RT-PCR analysis confirmed increased expression of uPA, uPAR, focal adhesion kinase (FAK), N-Cadherin and integrin subunits (e.g., α3, α5 and β1) in irradiated cells. Furthermore, we noticed a ∼2-fold increase in tyrosine phosphorylation of FAK in irradiated cells. Immunoprecipitation studies confirmed increased interaction of integrin β1 and FAK in irradiated cells. In addition, our results show that overexpression of uPAR in cancer cells can mimic radiation-induced activation of FAK signaling. Moreover, by inhibiting FAK phosphorylation, we were able to reduce the radiation-induced invasiveness of the cancer cells. In this vein, we studied the effect of siRNA-mediated knockdown of uPAR on cell migration and adhesion in irradiated and non-irradiated medulloblastoma cells. Downregulation of uPAR reduced the radiation-induced adhesion, migration and invasion of the irradiated cells, primarily by inhibiting phosphorylation of FAK, Paxillin and Rac-1/Cdc42. As observed from the immunoprecipitation studies, uPAR knockdown reduced interaction among the focal adhesion molecules, such as FAK, Paxillin and p130Cas, which are known to play key roles in cancer metastasis. Pretreatment with uPAR shRNA expressing construct reduced uPAR and phospho FAK expression levels in pre-established medulloblastoma in nude mice.

**Conclusion/Significance:**

Taken together, our results show that radiation enhances uPAR-mediated FAK signaling and by targeting uPAR we can inhibit radiation-activated cell adhesion and migration both *in vitro* and *in vivo*.

## Introduction

Medulloblastoma is the most common malignant brain tumor of childhood, which accounts up to 17–20% of intracranial pediatric tumors arising in the cerebellum and is often less diagnosed in adults [1], [2]. It has one of the highest rates of metastasis outside the central nervous system [3]–[6] and tends to spread hematogenously into bones, bone marrow, lymphatic nodes, liver, and lungs [7], [8]. When compared with other childhood tumors, the median survival rate of medulloblastoma is poor with a five-year survival rate of less than 50 percent. Surgical resection followed by craniospinal irradiation and chemotherapy has been the mainstay of therapy, which has improved the survival rate of patients. Despite these encouraging trends, sporadic late recurrences are well documented even after the most effective treatments [9], [10].

For decades, radiation therapy has been a mainstay in treating various cancers, and along with surgery and chemotherapy, radiation has been used as part of an integrated cancer therapy. The high-energy rays involved in radiotherapy keep a check on rapidly growing cancer cells by damaging cellular DNA, which leads to decreased tumor development [11]. However, a significant number of cancer recurrences have been reported in cancer patients treated with radiation. The recurrence, either at the primary tumor site (local) or a distant site/organ (metastasis), is not limited to medulloblastoma and has been reported in other brain tumors as well as breast, gastric [12], pancreatic [13], prostate [14] and lung cancers. Most of the recurrences for medulloblastoma emerge within 18 months of treatment [6] with a median survival period of 2 years and are predominant in the posterior fossa and extraneural metastases. The highly invasive ability of cells has been identified as a major reason for the low survival rate of patients with tumor recurrence. Both *in vitro* [15] and *in vivo* [16] studies have demonstrated that radiation enhances invasion and metastasis of cancer cells. Metastasis is a complex process largely dependent on cell adhesion to extracellular matrix (ECM)/basement membrane that triggers various signaling pathways, thereby allowing cancer cells to remodel the ECM, which is followed by cancer cell invasion, migration and establishment at a new site. Cell invasion is mediated by both extra- and intracellular factors and is dependent on the precise, dynamic interaction of various cell surface receptors with the ECM [17]–[19].

Among the cell surface receptors, integrins form a diverse group of transmembrane glycoproteins that facilitate an active interaction with other cell surface and ECM components, which coordinate the signaling cascades regulating cell adhesion, survival, and cytoskeleton organization [20]–[23]. uPAR is considered to be one of the transmembrane receptors that forms an active complex with integrins and plays a crucial role in activating integrin-mediated downstream signaling related to cell adhesion and migration [24]–[27]. More study is needed to better understand the role of uPAR (a GPI-anchored glycoprotein) in activating signals related to cell survival, adhesion and migration [26]. Reports suggest that uPAR interacts with integrins to confer specificity to the activated signaling pathway [28], [29]. In addition, uPAR forms a complex with ligands such as uPA and vitronectin that enhances the binding and assembly of various other ligands to integrins and subsequently activates downstream signaling [30]–[32]. However, considering the frequency of recurrence in patients who receive radiation therapy, we were primarily interested in determining the mechanism of radiation-induced cell adhesion and invasion in medulloblastoma. Further, given the role of the uPA/uPAR system in ECM proteolysis and its interaction with integrins to activate cell adhesion and the migration signaling cascade, we attempted to sensitize the cancer cell to radiation by targeting uPAR using RNA interference technology.

## Results

### Radiation reduces cell proliferation, but enhances cell adhesion and migration of medulloblastoma cells

MTT and trypan blue cell exclusion assays were performed to determine cell proliferation and viability in irradiated DAOY and D283 cells. After 36 hrs of radiation (7 Gy), the proliferation index of DAOY and D283 cells was reduced by 23% and 33%, respectively (Fig. 1A). Under the same experimental conditions, the percentage of viable cells was reduced by 17% and 25% in DAOY and D283 cells, respectively (Fig. 1B). Cell adhesion, matrigel and wound healing migration assays were carried out to determine the adhesive and migratory characters induced by radiation in DAOY and D283 cells. With the cell adhesion assay, we observed that radiation enhanced the adhesiveness of DAOY cells to collagen, fibronectin, vitronectin and matrigel by 38%, 50%, 67% and 120%, respectively as compared to non-irradiated cells (Fig. 1C). In D283 cells, radiation increased adhesion to collagen, fibronectin, vitronectin and matrigel by 38%, 61%, 97% and 80%, respectively (Fig. 1C and 1D). Among various ECM components tested, we noticed that radiation induced more adhesion to matrigel followed by fibronectin. Wound healing migration assay demonstrated that migration of irradiated DAOY cells was increased by ∼27% as compared to non-irradiated cells (Fig. 1E). We were unable to demonstrate the same in D283 cell line since these cells generally do not form a uniform monolayer, which is a key factor for performing the wound healing assay. In addition to enhanced cell adhesion and migration, we noticed that the matrigel invasion potential of the irradiated DAOY and D283 cells, when normalized with the percent proliferation and viability rate, was increased by 30% and 26% in these cell lines when compared to the respective non-irradiated cells (Fig. 1F).

**Figure 1:** Radiation reduced the survival rate but enhanced cell adhesion, migration and invasion of medulloblastoma cells. Cells were irradiated with 7 Gy and the effect of radiation on cell proliferation rate and viability was determined by (**A**) MTT assay and (**B**) trypan blue exclusion assay. Mean values (± S.D, *p*<0.001) from three independent experiments were represented graphically. (**C**) Radiation enhanced the adhesion of cells to ECM components. 24 hrs after irradiating the cells with 7 Gy, the cells were detached from the plates and an equal number of cells (irradiated [IR] and non-irradiated [non-IR]) were plated on a 96-well culture plate coated either with type-I collagen (5 µg/mL), fibronectin (2 µg/mL), vitronectin (2 µg/mL) and matrigel (50 µg/mL). After 1 hr (DAOY) or 3 hrs (D283), the cells that attached to collagen, fibronectin and vitronectin were stained with Hema-3 and visualized under a light microscope. The number of cells attached to matrigel was quantified by MTT assay. The number of cells attached to various ECM components was counted and graphically represented. Bars represent the mean ± S.D values from three different experiments (* and ** represents *p*<0.05 and *p*<0.005, respectively, compared to the respective non-irradiated cells in each group). (**D**) Represents the spreading of cells induced upon binding of IR and non-IR DAOY and D283 cells to ECM components. (**E**) Wound healing migration assay was carried out on DAOY cells. Distance migrated by non-IR and IR cells was compared and represented in the graph (mean ± S.D value from three independent experiments; * represents *p*<0.05 compared to non-irradiated DAOY cells). (**F**) Invasiveness of DAOY and D283 cells (with and without radiation) was quantified by counting the number of cells that invaded through matrigel. Results of five different experiments are represented (± S.D. value, ** *p*<0.05 compared to respective non-irradiated cells).

### Radiation enhances the expression of uPAR, integrins and phosphorylation of FAK

Various researchers have shown a direct correlation between increased levels of uPA/uPAR and the invasiveness of tumor cells. As such, we investigated the expression pattern of these proteases in irradiated cells. Zymography analysis using fibrinogen gels demonstrated that the activity of uPA was increased in a dose-dependent manner in the irradiated cells (Fig. 2A). The same was confirmed at the transcript level (Fig. 2B). uPA activity, as quantified by measuring the intensity of lytic zones on the zymography gels, was ∼4- and 3-fold higher in irradiated DAOY and D283 cells respectively, when compared to non-irradiated cells (Fig. 2C). Furthermore, the expression levels of uPAR both at the transcriptional and translational levels showed a dose-dependent increase in DAOY and D283 cells in response to radiation (Fig. 2A and 2B). Real time RT-PCR analysis of uPA and uPAR mRNA expression further strengthened the semi-quantitative RT-PCR results. Real time-PCR analysis showed a ∼3.9 and 4.2 fold increase in uPA and uPAR mRNA levels in irradiated DAOY cells, respectively, when compared to non-irradiated cells, whereas the uPA and uPAR levels were increased by 9 and 4.3 folds in irradiated D283 cells, respectively.

**Figure 2:** Radiation enhanced extracellular protease activity and aggressiveness of the cancer cells. (**A**) Medulloblastoma cells were irradiated with 7 Gy and serum starved for 24 hrs. The conditioned medium was collected and analyzed by SDS-PAGE gels either containing fibrinogen/plasminogen to determine the enzymatic activity of uPA. uPAR levels were detected in total cell lysates by immunoblotting with uPAR-specific antibodies. GAPDH antibody was used to confirm equal loading of the proteins in each lane. (**B**) Total RNA was isolated from the non-irradiated and irradiated cells, and transcript levels of uPA and uPAR were determined by RT-PCR analysis. (**C**) The enzymatic activity as determined by clear zone on the zymography gels were quantified by densitometry. Intensity of uPAR signals were quantified by densitometery and normalized with GAPDH. Graphical representation of values obtained from four independent experiments was presented with a mean ± S.D value, (*p<0.01 and ^#^ *p*<0.05 with reference to respective controls) (**D**) Translation modification of matrigel-invading cells (In) was compared between non-irradiated (non-IR) and irradiated (IR) cells. Total RNA was isolated from non-invading and matrigel-invading cells as described in Materials and Methods. RT-PCR analysis was carried out for transcript levels of integrin subunits, uPAR, uPA, N-Cadherin and FAK were determined using specific primers. GAPDH was used as a control. (**E**) The amplicon intensity was quantified and represented. Results from two different experiments are represented (± S.D. value, * *p*<0.05 and # *p*<0.01 with reference to non-invading controls).

Our next set of experiments were targeted to determine integrin expression levels in the cells irradiated with 7 Gy since these molecules were considered to directly effect cell adhesion and indirectly effect the signaling cascade related to cell adhesion and migration, especially through FAK-mediated signaling. Using RT-PCR analysis, we compared the expression pattern of integrin sub units (α1-6 and β1-6) in irradiated and non-irradiated cells. We observed that the transcript levels of integrin α3, α5, β1 and β6 subunits were significantly elevated upon radiation in DAOY cells. In D283 cells, integrin α1, α3, α4, α5 and β1 subunits were increased upon radiation (Fig. S1A). The increase in uPA proteolytic activity and integrin expression in irradiated cells directed us to examine the transitional character of irradiated cells invading through matrigel. Hence, we carried out a matrigel invasion assay of non-irradiated and irradiated cells and isolated the total RNA from non-invaded cells and matrigel-invaded cells. RT-PCR analysis showed a clear demarcation of the aggressive behavior of matrigel-invading cells as compared to non-invading cells; this was more prominent in irradiated cells (Fig. 2D). Comparison of non-invading control cells and irradiated invading cells showed a significant increase of ∼2-fold in uPA, uPAR and FAK expression in irradiated DAOY and D283 cells. In addition, a ∼3-fold increase was observed in the transcripts level of N-Cadherin and integrin β1 in irradiated DAOY and D283 cells (Fig. 2E).

The elevated expression of membrane associated molecules such as uPAR and integrins, directed us to examine the downstream signaling cascade induced by radiation. The role of uPAR/integrin β1 in activating FAK signaling has been described in various cancer types under *in vitro* and *in vivo* conditions [28]. Since there was an increase in uPAR and integrin β1 levels in irradiated medulloblastoma cells, we analyzed the activation of FAK and the subsequent signaling cascade, which lead to enhanced cell adhesion and migration. We observed a ∼2-fold increase in the phosphorylation of FAK at 397 tyrosine residue in irradiated DAOY and D283 cells as compared to respective non-radiated cells (Fig. S1B). The phosphorylation levels of Src and Paxillin were also increased in irradiated cells (Fig. S1B). However, our attempts to detect the effect of irradiation on tyrosine phosphorylation of FAK at 576/577 and 925 residues were not consistent (data not shown).

To support our contention that radiation-induced uPAR/integrin β1 activates the FAK signaling cascade, we carried out a co-immunoprecipitation assay. When the co-immunoprecipitates of uPAR were analyzed by immunoblotting with integrin β1 antibody, we noticed that the association of uPAR with integrin β1 was increased in irradiated cells as compared to control cells (Fig. 3A). Subsequently, when immunoprecipitates of integrin β1 were analyzed by immunoblotting with uPAR and phospho FAK (Y397) antibodies, we observed that the interaction of integrin β1 with uPAR and phospho FAK was high in irradiated cells, indicating that radiation enhanced both the interaction and activation of FAK signaling associated with ligation of integrin β1 (Fig. 3B). Furthermore, an immunofluorescence assay confirmed the co-localization of uPAR and integrin β1 at the migratory front of the irradiated cells (Fig. 3C).

**Figure 3:** Radiation induced uPAR/integrin β1/FAK interaction led to activation of FAK/Src/Rac signaling. Co-immunoprecipitation assay was carried out to determine the interaction of uPAR with integrin ββ1. Cells were irradiated and detached from the culture plate using a cell stripper solution. Total cell lysates were immunoprecipitated with either uPAR or integrin β1. (**A**) Immunoprecipitates of uPAR were analyzed by immunoblotting with integrin β1 and uPA antibodies. (**B**) Immunoprecipitates of uPAR/integrin β1 were analyzed by western blotting with uPAR, FAK and pFAK (Y397). (**C**) Immunofluorescence assay was used to detect the localization of uPAR/integrin β1 in irradiated and non-irradiated cells. Cells seeded on 2-well chamber slides were irradiated with 7 Gy and incubated for 24 hrs. The cells were incubated with uPAR and integrin β1 antibodies followed by incubation with species-specific Alexa Fluor secondary antibodies. Immunofluorescence assay demonstrates the co-localization (yellow color) of uPAR and integrin β1 at the migratory front of irradiated cells.

### Activation of FAK-mediated signaling in irradiated cells promotes migration

To elucidate the molecular mechanism by which radiation induces cell adhesion and invasion, we transfected full length uPAR (FL-uPAR) expressing plasmid into DAOY and D283 and examined whether we could mimic the radiation-induced uPAR signaling cascade. Overexpression of FL-uPAR in DAOY cells enhanced the phosphorylation of FAK, Paxillin and Rac-1/Cdc42 in DAOY and D283 cells (Fig. 4A). In DAOY cells, the phosphorylation of FAK, Paxillin and Rac-1/Cdc42 was increased by 70%, 72% and 76%, respectively. In D283 cells, FL-uPAR expression has increased the phosphorylation of FAK, Paxillin and Rac-1/Cdc42 by 52%, 56% and 66%, respectively (Fig. S2A). The cumulative effect of radiation and FL-uPAR expression together was shown to increase the invasive ability (see Fig. 4C) as well as the activation of FAK, Paxillin and Rac-1/Cdc42 when compared to either FL-uPAR transfection or radiation alone (Fig. 4A). The phosphorylation of FAK at Y397 was increased by ∼2.6- and 2.3-fold in irradiated FL-uPAR-transfected DAOY and D283 cells, respectively compared to non-irradiated cells (Fig. S2A). Although we were unable to detect the phosphorylated form of p130Cas, we did observe an increase in the basal expression levels of the p130Cas protein in FL-uPAR-transfected cells.

**Figure 4:** uPAR overexpression enhances FAK signaling and cell invasion in medulloblastoma cells. (**A**) DAOY and D283 cells were transiently transfected with full length uPAR (FL-uPAR) for 48 hrs. Transfected cells were either irradiated with 7 Gy or non-irradiated and incubated for another 24 hrs. Total cell lysates were immunoblotted with the indicated antibodies. (**B**) Inhibiting FAK phosphorylation reduced the radiation-induced activation of FAK signaling cascade and cell invasion. DAOY and D283 cells were treated with or without FAK inhibitor for 2 hrs and then subjected to radiation and incubated for another 24 hrs. Phosphorylation levels of FAK (Y397) and downstream signal molecules, such as Paxillin and Rac-1/Cdc42, were confirmed by immunoblotting the total cell lysates with specific antibodies. (**C**) FL-uPAR-transfected and/or FAK inhibited cells (either irradiated or non-irradiated) were subjected to matrigel invasion assay to determine the invasive potential of uPAR overexpression in cancer cells. The number of cells invaded per each treatment was counted and graphically presented. Results from three different experiments were complied and represented with a ± S.D mean value, *p*<0.05.

To further evaluate whether radiation-induced cell adhesion and invasion is associated with FAK-mediated signaling, we examined the effect of molecules involved in migration by inhibiting tyrosine phosphorylation of FAK at 397. Inhibition of FAK phosphorylation using FAK inhibitor has significantly reduced the radiation-induced activation of FAK by 60% and 66% in DAOY and D283 cells, respectively (Fig. 4B and Fig. S2B). In addition, inhibition of FAK phosphorylation has reduced the phosphorylation of the downstream signaling molecules such as, Paxillin by 54% and 71% and Rac-1/Cdc42 by 45% and 66% in DAOY and D283 cells, respectively (Fig. S2B). Moreover, inhibition of FAK has also reduced the expression of integrin β1, which suggests that the inhibition of FAK phosphorylation affected cell adhesion, which in turn might have affected the expression of integrin β1. Further, the combination of FL-uPAR transfection and radiation increased matrigel invasion of both DAOY and D283 cells by ∼2-fold (Fig. 4C). Inhibition of FAK phosphorylation reduced the matrigel invasion potential of irradiated cells and significantly reduced the invasive ability of irradiated and FL-uPAR-expressing cells (Fig. 4C).

### shRNA-mediated uPAR downregulation inhibits radiation-induced cell adhesion and migration of medulloblastoma cells

Given the fact that uPAR plays a key role in the activation of ECM proteolysis and initiation of the signaling cascade related to cell survival, adhesion, migration and invasion, we next determined the potential of siRNA-mediated downregulation of uPAR in sensitizing the radiation-induced cell adhesion and migration associated with activation of integrin β1 and FAK signaling. shRNA plasmid transfection resulted in downregulation of uPAR both at the transcript and translational levels in DOAY and D283 cells (Fig. 5A1 and 5A2). Moreover, siRNA-mediated targeting uPAR using the siRNA-expressing plasmid pU reduced the transcript levels of FAK and integrin β1 in DAOY and D283 cells (Fig. 5A1). Further, RT-PCR analysis showed that downregulation of uPAR reduced the radiation-induced expression of integrin β1 by 56% and 53% in DAOY and D283 cells, respectively (Fig. 5B). The transcripts levels of FAK were reduced by 47% and 44% in DAOY and D283 cells, respectively. With the reduction of these key molecules, we initially examined the effect of pU transfection on the adhesion of cells to various ECM components. DAOY cells transfected with pU followed by irradiation showed a reduction in cell adhesion to collagen, fibronectin and vitronectin by 48%, 71% and 64%, respectively. Adhesion to collagen, fibronectin and vitronectin was reduced by 43%, 45% and 62%, respectively in pU-transfected and irradiated D283 cells (Fig. 5C).

**Figure 5:** siRNA-mediated downregulation of uPAR reduced radiation-induced cell adhesion, invasion and migration. A plasmid expressing siRNA against the uPAR gene (pU) was transiently transfected into DAOY and D283 cells. The efficiency of uPAR downregulation was confirmed by RT-PCR analysis using specific primers. (**A1**) After 36 hrs of transfection, the cells were either irradiated with 7 Gy or non-irradiated and incubated for another 24 hrs before total RNA was isolated. RT-PCR analysis was carried out to determine the effect of uPAR knockdown on the transcriptional levels of uPAR, integrin β1 and FAK. GAPDH was used as a loading control. (**A2**) Western analysis of the total cell lysates extracted from uPAR knockdown cells (with and with radiation) with uPAR and GAPDH antibodies. (**B**) Amplicon intensity was measured using densitometry. Data shown are the mean of three different experiments and the bars are ± S.D. (* *p*<0.05 with IR and # *p*<0.01 with control). (**C**) The effect of uPAR downregulation and radiation on the cells adhesive properties was determined by plating cells onto ECM component-coated plates. 1×10^4^ cells were allowed to adhere to plates coated (**a**) type-I collagen, (**b**) fibronectin or (**c**) vitronectin. After allowing the cells to attach for 1 hr (DAOY) or 3 hrs (D283), the wells were washed and stained with Hema-3. The number of adhered cells was counted under a light microscope and quantified data from three different experiments are represented graphically (mean ± S.D., * represents *p* value of <0.01).

As we expected, knockdown of uPAR significantly reduced matrigel invasion and migration of irradiated and non-irradiated DAOY and D283 cells as compared to non-transfected cells or cells transfected with pSV (scrambled vector). Moreover, pU reduced invasion of the irradiated cells by 62% in DAOY cells and 69% in D283 cells as compared to non-irradiated cells (Fig. 6A and 6B). The wound healing migration assay carried out with DAOY cells showed that uPAR knockdown reduced the ability of cells to migrate towards each other by ∼50% as compared to the control cells (Fig. 6C and D).

**Figure 6:** Knockdown of uPAR reduced radiation-induced cell invasion and migration. Knockdown of uPAR inhibited radiation-enhanced cell adhesion, invasion and migration by blocking uPAR/integrin β1/FAK interactions. After 48 hrs of pU transfection, the cells were either irradiated or non-irradiated before analysis for cell adhesion, invasion and migration potential. Cells were detached from the culture plate using cell stripper solution for further analysis. (**A**) 2×10^5^ cells were plated on matrigel-coated transwell inserts and incubated for 24 hrs to determine the invasive potential of irradiated and non-irradiated pU-transfected cancer cells. The matrigel-invading cells were stained with Hema-3 and visualized under a light microscope. (**B**) The number of invading cells was counted from five different fields and quantified; a comparison between various treatments is represented graphically. Percent cell invasion was measured from the mean obtained from three independent experiments and values shown are the mean ± S.D (* *p*<0.005 with reference to irradiated control). (**C**) Wound healing migration assay was carried out to determine the migratory ability of irradiated and non-irradiated pU-transfected cells. Transfected cells were grown until a monolayer formed and then a scratch was made using a 200-µL pipette tip. After thorough washing with PBS, the cells were either left non-irradiated or irradiated with 7 Gy. The distance migrated by the cells was monitored over a period of time by observation under a light microscope. (**D**) This was further quantified and data are represented graphically as a mean of three different experiments with ± S.D (* represents *p*<0.05).

### uPAR knockdown blocks radiation-induced integrin β1/FAK signaling in medulloblastoma cells

We determined the effect of uPAR downregulation on radiation-induced activation of FAK signaling. Western blot analysis showed that downregulation of uPAR in DAOY and D283 cells effectively reduced the expression of radiation-induced levels of integrin β1 (Fig. 7A). Further, we noticed significant reductions in phosphorylation of FAK at Y397 in pU-transfected DAOY and D283 cells, respectively (Fig. 7A). We next analyzed the signaling molecules known to be activated upon FAK phosphorylation, and we observed that uPAR knockdown reduced the phosphorylation of Src (Y417), Paxillin, Rac-1/Cdc42 in both irradiated and non-irradiated cells (Fig. 7A).

**Figure 7:** uPAR knockdown reduces radiation-induced FAK signaling cascade by disrupting the interaction of focal adhesion molecules. (**A**) Total cell lysates extracted from uPAR knockdown cells (either irradiated or non-irradiated) were analyzed by immunoblotting with integrin β1, phospho FAK (Y397), Paxillin, Rac-1/Cdc42 and p130Cas. GAPDH was used as a loading control. Radiation enhanced tyrosine phosphorylation of FAK was reduced by inhibiting the interaction of uPAR and integrin β1 in pU-transfected cells. Total cell lysates were subjected to immunoprecipitation with either integrin β1 or FAK. (**B**) The immunoprecipitates of integrin β1 were analyzed by western blotting with antibodies specific for uPAR and FAK. (**C**) The co-immunoprecipitates of FAK were analyzed by western blotting with antibodies specific for phospho FAK, Paxillin and p130CAS.

We also examined the effect of uPAR knockdown on the interaction/activation of integrin β1 and FAK by co-immunoprecipitating the total cell lysate either with integrin β1 or FAK, followed by western blot analysis with antibodies for uPAR, FAK, phospho FAK and p130Cas (Fig. 7B). uPAR downregulation dramatically reduced the interaction of integrin β1 with uPAR in both non-irradiated and irradiated cells (Fig. 7B). When immunoprecipitates of FAK were analyzed by western blotting with phospho FAK and p130Cas, we noticed that pU transfection reduced the phosphorylation levels of FAK and the interaction of FAK with p130Cas protein (Fig. 7C). We even observed a similar effect in the cells where phosphorylation of FAK was inhibited (data not shown). We did not notice any specific interaction of FAK with Rac-1 or its active form. However, we did observe that the interaction of p130Cas and FAK was high in irradiated cells as compared to non-irradiated cells, and this interaction was reduced in pU-transfected cells.

### uPAR treatment prior to radiation significantly inhibits the tumor development

Our *in vitro* studies inferred that knockdown of uPAR prior to irradiation has significantly inhibited the radiation induced phosphorylation of FAK and subsequent downstream signaling molecules. Therefore, the effect of shRNA expressing plasmid on pre-established medulloblastoma in nude mice was studied. Generally, after 5–6 weeks of tumor cells injection we noticed that the control animals started to loose weight and showed certain behavioral symptoms. Therefore, we euthanized all the animals at this particular time period, irrespective of the fact that the irradiation and pU treated mice were showing no obvious weight loss or other symptoms. Hematoxylin and eosin (H&E) staining of the paraffin embedded brain tissue section confirmed the presence of prominent regions of proliferating tumor cells in the control and pSV treated tumor compared to pU treated tumors. H&E stained tumor sections showed that pU treatment has reduced the tumor volume by nearly 49% compared to the control mice. Further, the radiation treated intracranial tumor showed less (20%) dense tumor cells compared to the non-irradiated tumors. Moreover, treatment of the tumors with pU prior to irradiation showed a prominent inhibition in tumor cell growth by nearly 85% when compared to the controls (Fig. 8A and B). Considering the invasive fronts of the tumor and the metastasized tumor bodies as migratory/invasive index, we observed that tumors treated with irradiation alone increased the number of metastasized tumor bodies at the invasive fronts of the primary tumor area when compared to non-irradiated tumors. However, the tumors treated with pU alone or along with irradiation showed a reduced metastasized tumor bodies when compared to tumors treated with pSV or control (Fig. 8C). Further, to determine the effect of irradiation and pU treatment on uPAR and FAK expression levels in intracranial tumors, we carried out immuno-histochemical (IHC) analysis of paraffin embedded brain sections. We observed that uPAR and phospho FAK (Y397) staining were high in the irradiated brain sections compared to control brain sections (Fig. S3). Enhanced staining intensity observed on irradiated brain tissue sections is indicative of radiation induced expression of uPAR and phosphorylation of FAK in intracranial tumors. Moreover co-relating with *in vitro* studies, pU treated tumors has prominently reduced the expression levels of uPAR and phospho FAK compared to controls or tumors treated with pSV.

**Figure 8:** Effect of uPAR siRNA expressing plasmid treatment prior to radiation on pre-established intracranial tumor. (**A**). Hematoxylin and eosin (H&E) staining performed on the paraffin embedded tissue sections of pre-established tumors from untreated and mice treated with either pU or pSV followed by with or without radiation. Experiments were carried out on five animals in each group. (**B**) Tumor volumes were quantified and represented graphically. (n = 5 with mean ± S.D; *p<0.05 with reference to non-irradiated control mice. (**C**) H&E staining of the brain section was carried out and representative pictures of brain sections showing the migratory fronts and metastatic bodies from control, pSV and pU (with and without radiation) treated mice are shown.

## Discussion

The advent of various chemotherapeutic drugs and molecular marker-based therapeutics has not replaced radiation therapy as a mainstay of cancer treatment. Radiotherapy remains the single most effective treatment for various cancers, including medulloblastoma. However, after successful surgical resection followed by craniospinal radiation, it has been well documented that this treatment module induces medulloblastoma recurrence [2], [6], [33], [34]. Although radiation decreases the proliferation rate of cancer cells, several *in vitro* studies have demonstrated that sublethal doses of radiation resulted in increased invasiveness of cancer cells [15], [35]–[38]. Moreover, laboratory studies have demonstrated that local radiotherapy administered to primary tumors enhanced the metastatic growth of the tumors [16], [39], [40]. Overall, it is clear that the adjuvant radiotherapy used for local tumor growth control increases the probability of developing distant metastasis in cancer patients. However, the molecular mechanism of this radiation-induced cancer metastasis is not yet completely understood.

In the present study, we compared the cell invasion, adhesion and migration potential of irradiated and non-irradiated cancer cells, and we made an attempt to understand the molecular mechanisms underlying radiation-induced cell adhesion and invasion of medulloblastoma cells under *in vitro* conditions. Our studies have shown that radiation reduced the proliferation and the viability rate of both DAOY and D283 cells, indicating that radiation keeps a check on cancer cell cycle progression. However, radiation-induced recurrence at the primary site or at a distant site (metastatic tumor) is more related to the enhanced migratory properties of the cancer cells. The three-step hypothesis for tumor cell invasion was proposed, which includes 1) adhesion of cell to the ECM, 2) degradation of the ECM by cellular proteases, and 3) migration/invasion through the ECM [41]–[43]. Therefore, we further examined cell adhesion, invasion and migration induced by radiation. Indeed, we observed that irradiated cells had increased adhesion to collagen, fibronectin, vitronectin and matrigel, as well as the potential to invade the matrigel. Similar observations have been reported on radiation-enhanced cell invasion, migration and adhesion to various ECM in lung [44], [45] and hepatoceullar carcinoma [35]. Increased cell invasion is generally reported to be associated with proteolytic activity of various extracellular proteases secreted by cancer cells. The roles of the uPA system (uPA and uPAR) in ECM remodeling and cancer cell invasion and migration have been well characterized and are associated with the invasive and migratory characteristics of irradiated cancer cells [46]–[48]. The results of the present study confirmed that radiation induced the expression and activity of uPA (a serine protease). Given the fact that cells tend to constantly vary their phenotype from epithelial to mesenchymal during the process of invasion [49]–[51], we made an attempt to determine the radiation-induced variation of the molecules known for their functional relevance with cancer cell invasion. Furthermore, radiation-induced invasiveness and migration have been reported to be associated with enhanced expression of epithelial–mesenchymal transition (EMT)-related molecules [15], [44]. In this context, our attempts to differentiate non-invading from invading cells demonstrate that the latter tend to show increased expression of uPAR, uPA, N-Cadherin and various integrin subunits. Increased expression of these molecules in the irradiated cells suggests that the aggressiveness and EMT of the matrigel-invading irradiated cells is more than that of the invading non-irradiated cells. Earlier studies have shown that the metastatic process involves the interaction of cell surface molecules and their binding ligands to ECM as well as activation of associated signaling pathways [52]–[54]. Similarly, in the present study, we noticed increased expression of various integrin subunits, uPAR and FAK, suggesting that these molecules might play an important role either by directly aiding in cell adhesion and invasion or by activating signaling processes related to cell motility. Collectively, our studies show that radiation reduces the rate of cell proliferation, but enhances cell adhesion, migration and invasion of the cancer cells *in vitro*, leading to an increased metastatic potential of the irradiated medulloblastoma cells.

Among the integrin subunits, we noticed that the expression of integrin β1, α3 and α5 subunits were commonly increased with radiation in both DAOY and D283 cells. Our additional studies were focused on integrin subunit β1, as several researchers have demonstrated that uPAR activates various signaling cascades through its interaction with an integrin heterodimer comprising the β1 subunit [29], [55], [56]. Moreover, among various integrin heterodimers, subunit β1 containing integrins were reported to play critical roles in recruiting and activating FAK [57], [58]. In addition, uPAR-integrin β1 interactions are frequently associated with the activation of signals favoring tumor growth, possibly through activation of the FAK/Src signaling pathways [28], [29], [59]–[61]. Jung [44] showed that radiation-enhanced cell adhesion and invasion are associated with increased expression and/or activation of various focal adhesion molecules, such as FAK and Paxillin, which are critical mediators of integrin-activating signaling to promote cell migration. Indeed, our results show that radiation induced activation of FAK by phosphorylating tyrosine residue at 397 Src at Y416 and Paxillin at Y118. Moreover, the increased phosphorylated forms of Rac-1/Cdc42 in the irradiated cells directed us to confirm that integrin-mediated cell mobility was induced by radiation.

Activation of Rac-1 is considered as an important step in integrin signaling [62], [63]. Previous reports also suggested that the interaction of uPAR with integrin β1 activates Rac-1 through an enhanced FAK/Src signaling pathway during the process of tumor cell invasion [29]. Furthermore, immunoprecipitation studies have shown that interaction of integrin β1 with uPAR was significantly higher in irradiated cells. When we tested the co-immunoprecipitates of integrin β1 with total and phospho FAK, we noticed that phospho FAK (Y397) was immunoprecipitated with integrin β1 to a significantly higher level in irradiated cells as compared to non-irradiated cells. This finding suggests that the uPAR/integrin β1 interaction induced by radiation could mediate the tyrosine phosphorylation of FAK, which leads to the activation of signals that enhance cell adhesion and invasion. To support our finding, we inhibited tyrosine phosphorylation of FAK at 397 and determined the downstream effects in irradiated cells. As expected, we noticed that the inhibition of FAK activation decreased Rac-1 activation, which in turn, inhibited the radiation-induced invasion potential of cancer cells. Recent reports have also shown that phosphorylation of FAK at Tyr 397 correlated with tumor stage and the migratory and invasive abilities of hepatocellular carcinoma [64]. The increased phosphorylation levels of FAK resulting from over expressing FL-uPAR in cancer cells provides further evidence of radiation-induced activation of FAK being mediated by uPAR. The cumulative effect of FL-uPAR expression in irradiated cells as well as matrigel invasive ability and phosphorylation of FAK, Src/Paxillin and Rac-1/Cdc42 strengthen our inference that radiation-induced uPAR activates FAK signaling to promote cancer cell invasion and adhesion. Recently, it has been demonstrated that FAK-mediated activation of cell migration and adhesion involves focal adhesion turnover dynamics as well as cytoskeleton polymerization of various molecules, such as vincullin, α-actinin and talin [57], [65], [66]. Collectively, these data indicate that uPAR expression and activation of FAK are essential for the increased cell invasion and migration induced by radiation. Taken together, our studies indicate that radiation-induced uPAR/integrin β1 interaction activates FAK signaling, thereby leading to enhanced cell invasion and migration in medulloblastoma cells. We conclude that FAK signaling activated by radiation ultimately leads to enhanced cell adhesion and invasion.

The involvement of uPAR in the proteolysis of ECM and the activation of cellular signaling through its interaction with integrins and/or other ligands is well established [67]–[70]. Previous reports from our lab and others have suggested that knockdown of uPAR significantly reduced the invasive potential of cancer cells under *in vitro* and *in vivo* conditions. Therefore, we further attempted to knockdown uPAR using siRNA and then determined the effect on radiation-induced cell adhesion, invasion and associated signaling pathway(s). Similar to earlier reports, the present study confirmed that depletion of uPAR inhibited matrigel invasion, adhesion to ECM components, and migratory potential of both non-irradiated and irradiated cells *in vitro*. The decrease in the phosphorylation levels of FAK, Src, Paxillin and Rac-1/Cdc42 in irradiated and non-irradiated cells confirmed that the downregulation of uPAR impaired the radiation-induced activation of FAK/Src signaling, which might have led to a reduced invasive potential of pU-transfected cells. The immunoprecipitation assays provided further evidence that showed the depletion of uPAR from the cell surface not only reduced the uPAR/integrin β1 complex but also the interaction of FAK with Paxillin and p130Cas (adapter focal adhesion molecules). Both Paxillin and p130Cas are the main phosphorylation targets of the FAK/Src signaling complex necessary for cell motility and adhesion [71], [72]. In the present study, radiation induced the interaction of FAK with p130Cas, suggesting that the radiation not only induced FAK signaling but also initiated FAK to play a role in recruiting p130Cas to activate cell adhesion and migration. Earlier reports have also suggested that uPAR interacts with integrin complexes to promote the interaction of FAK with p130Cas [73] and p130Cas–CrkII signaling complex to activate Rac, thereby resulting in a Rac-mediated cell motility and invasion [74]. Collectively, the results of the present study demonstrate that the knockdown of uPAR reduced uPAR/integrin β1 complex formation, which can be co-related to decreased coordination between various focal adhesion molecules as determined by co-immunoprecipitation of FAK and p130Cas. As observed in the present study, the decrease in p130Cas binding to FAK has been reported to abolish both phosphorylation of p130Cas by FAK/Src complex and stimulation of cell migration by FAK [75].

Nevertheless, we suspect that the reduction of uPAR prior to radiation could retard the process of radiation-induced invasion by inhibiting the activation of migratory signals as well as by disrupting the coordination of focal adhesion molecules during the process of cell adhesion and migration. Our preliminary data on the effect of uPAR inhibition disrupting focal adhesion molecules provide a better understanding of the role of uPAR in coordinating the focal adhesion molecules in the process of cell motility. Here, we have demonstrated that downregulation of uPAR not only reduced medulloblastoma cell invasive and migratory capacity but also has the potential to sensitize the tumor for radiation therapy by disrupting the uPAR/integrin/FAK complex essential for cell invasion and migration.

## Materials and Methods

### Ethics Statement

The Institutional Animal Care and Use Committee of the University of Illinois College of Medicine at Peoria, Peoria, IL, USA, approved all surgical interventions and post-operative animal care. The consent was written and approved. The approved protocol number is 857, dated May 27, 2009 and renewed on May 17, 2010.

### Cell lines, chemical reagents, radiation and transfection conditions

Medulloblastoma cell lines (DAOY and D283) were obtained from ATTC (American Type Culture Collection, Manassas, VA). DAOY cells were maintained in advanced MEM medium supplemented with 5% fetal serum albumin (Invitrogen Corporation, Carlsbad, CA), 1% L-glutamine, 50 units/mL penicillin and 50 µg/mL streptomycin (Life Technologies, Inc., Frederick, MD). D283 cells were maintained in improved MEM medium supplemented with 10% fetal bovine serum (FBS), penicillin and streptomycin. Both the cell lines were maintained in a 37°C incubator in a 5% CO_2_ humidified atmosphere. We used the following antibodies for the present study: uPAR, integrin β1, focal adhesion kinase (FAK), phospho FAK (Y397), and glyceraldehyde-3-phosphate dehydrogenase (GAPDH) (Santa Cruz Biotechnology, Santa Cruz, CA); Paxillin, phospho Paxillin, phospho Src (Y417 and Y527), phospho Rac-1/Cdc42, p130Cas, Talin-1 (Cell Signaling Technology Inc., Beverly, MA); and Rac-1 (BD Transduction Laboratories, San Jose, CA). Species-specific secondary antibodies conjugated to HRP, Alexa Fluor 488, and Alexa Fluor 595 (Santa Cruz Biotechnology, Santa Cruz, CA) were used in this study. The FAK inhibitor 14 (1,2,4,5-Benzenetetramine tetrahydrochloride) was obtained from Tocris Bioscience (Ellisville, MO). All transfections were carried out using FuGene HD transfection reagent as per the manufacturer's protocol (Roche Applied Science, Madison, WI). Cells were transfected either with plasmid-expressing siRNA against uPAR (pU) [76], [77] or plasmid-expressing full length human cDNA clone of uPAR (FL-uPAR) (SC319092, OriGene Technologies, Inc. Rockville, MD). For radiation treatment, cells were irradiated with different doses of radiation using a RS 2000 Biological Irradiator (Rad Source Technologies Inc., Boca Raton, FL). Cells were grown to nearly 70–80% confluence and then treated with FAK inhibitor (5 µM) for 1–2 hrs followed by irradiation at 7 Gy. For combination treatment (transfection and radiation), cells were irradiated 36 hrs after transfection and incubated for another 16–20 hrs before further analysis.

### Cell proliferation and viability assays

Cell growth rate was determined using the MTT assay ([3-(4, 5-dimethylthiazol-2-yl)-2, 5-diphenyltetrazolium bromide]; Sigma Aldrich, St. Louis, MO) as described previously [78]. Briefly, 10 µL of MTT reagent was added to each well containing cells which were either non-radiated or irradiated; and incubated at 37°C for 4 hrs. DMSO was added to each well to dissolve the formazan crystals and absorbance was measured at 550 nm using a microplate reader (Benchmark, Bio-Rad, Hercules, CA). To determine the effect of radiation on cell viability, we carried out the trypan blue exclusion assay. After 24 hrs of radiation, the cells were suspended in equal volume of trypan blue stain (0.4% w/v) and incubated for 5 min. Then, we counted the cells using the Countess Automated Cell Counter (Invitrogen, CA).

### Cell adhesion, matrigel invasion and wound healing migration assays

For the cell adhesion assay, cells (1×10^4^) (either irradiated or non-irradiated) were plated on a 96-well plate previously coated with type-I collagen (5 µg/mL), fibronectin (2 µg/mL), matrigel (100 µg/mL), vitronectin (2 µg/mL) or bovine serum albumin (100 µg/mL). After 1 hr (DAOY) or 3 hrs (D283), the attached cells were washed with PBS three times. Cells that were adhered to the ECM components were quantified either by MTT assay (matrigel-coated plates) or by staining with Hema-3 stain (Fisher Diagnostics, VA). Images of the stained cells from different fields were taken under a light microscope (Olympus IX-71).

Matrigel invasion was carried out as described previously [78]. Briefly, 2×10^5^ cells (either non-irradiated or irradiated) treated with or without FAK inhibitor were plated on matrigel-coated transwell inserts and placed in a 12-well plate containing serum medium. For transfection experiments, cells which were either transfected alone or treated in combination with radiation were plated onto matrigel-coated transwell inserts. After overnight incubation, lower invaded cells were stained with Hema-3 stain. Images of the invaded cells were taken under a light microscope (Olympus IX-71, Minneapolis, MN). For wound healing migration assay, the cells (either irradiated or non-irradiated and transfected) were grown to full confluence to form a monolayer and a scratch was made as described previously [44], and the cells were allowed to migrate towards each other. By carefully monitoring under a light microscope, the distance migrated by the cells over the indicated time periods was measured and quantified.

### Reverse transcription polymerase chain reaction (PCR) and Real Time (RT)-PCR

Total RNA was extracted from transfected cells (either irradiated or non-irradiated and with or without transfection) using TRIZOL reagent (Invitrogen, CA) as per standard protocol. RNA (1 µg) was used as a template for reverse transcription reaction (Roche Applied Science, Indianapolis, IN), followed by PCR analysis using specific primers for uPA, uPAR, integrin subunits α1-6 and β1-6, FAK, N-Cadherin and GAPDH (Table S1). The amplified products were analyzed on an agarose gel. Real time PCR was carried out using FastStart SYBR Green master mix (Roche Applied Science, Madison, WI) on an BioRad IQCycler Detection system (Bio-Rad, Hercules, CA) as per the manufacturers instruction. The relative mRNA expression levels of uPA and uPAR were calculated based on the mean GAPDH expression levels of the representative sample.

### Zymography, immunoblotting and immunoprecipitation assay

Conditioned medium collected from the cells (either irradiated or non-irradiated and with or without transfection) was electrophoresed under non-reducing conditions on SDS-PAGE gels containing fibrinogen/plasminogen to detect the activity of uPA, as described previously [28], [29]. For western analysis, equal amounts of protein fractionated on SDS-PAGE was immunoblotted with primary antibody and subsequently incubated with species-specific, horseradish peroxidase-conjugated secondary antibodies (Santa Cruz Biotechnology, CA). Signals were detected using the ECL western blotting detection system (Pierce, Rockford, IL). Immunoprecipitation assays were carried out by incubating a minimum of 800 µg total cell lysate with antibody for 3 hrs at room temperature or overnight at 4°C on a rotating shaker. Protein A/G agarose beads (Miltenyi Biotec, Auburn, CA) were added to the above complex and incubated for either 30 min on ice or overnight at 4°C. These beads were passed through µM columns and immunoprecipitates were eluted as per the manufacturer's instructions. The immunoprecipitates were immunoblotted with primary antibodies.

### Immunofluorescence

For immunofluorescence, cells grown in two-well chamber slides were washed with PBS, fixed, permeabilized with ice-cold methanol and blocked with 2% BSA in PBS. Cells were incubated with primary antibodies for either 2 hrs at room temperature or overnight at 4°C, washed with PBS, and incubated with fluorescent-labeled, species-specific secondary antibodies (Alexa Fluor®) for 1 hr at room temperature. Before mounting, the slides were washed with PBS and incubated for a brief period with DAPI for nuclear staining and analyzed with a microscope (Olympus BX61 Fluoview, Minneapolis, MN)

### *In vivo* studies

DAOY cells (1×10^5^) were injected intracerebrally into nude mice as previously described [78]. After allowing the tumor to establish (8 to 10 days), the animals were separated into different treatment groups (a minimum of five in each group). Alzet osmotic pumps (model 2001, Alzet Osmotic Pumps, Cupertino, CA) were implanted into the animals for plasmid delivery (6–8 mg/kg body weight) as described previously [77]. A week after plasmid delivery, animals were give radiation treatment (7 Gy). Based on their performance and behavior, the animals were euthanized as appropriate. Mice were sacrificed by intracardiac perfusion with PBS followed by 10% buffered formaldehyde. The brains were excised from the animals, fixed in 10% buffered formaldehyde and embedded in paraffin. Tissue sections were subjected to hematoxylin and eosin (H&E) staining and immunohistochemistry analysis for the detection of tumor cells/volume and protein expression in the tumor, respectively, as described previously [78].

### Statistical analysis

All the western blot and RT-PCR data were quantified by measuring the band/signal intensity by densitometry analysis using ImageJ software (National Institutes of Health). Results were analyzed using the one-way analysis of variance (ANOVA) either followed by Bonferroni's post hoc test (multiple comparison tests, using GraphPad Prism version 3.02) or *t-*test to assess statistical significance. The difference was considered statistically significant with a *p* value either less than 0.005, 0.05 or 0.01.

## Supporting Information

Figure S1 Radiation induces expression of integrins and activates FAK signaling molecules. (A) Total RNA isolated from non-irradiated and irradiated DAOY and D283 cells was subjected to RT-PCR analysis using specific primers for integrin subunits. Under our experimental conditions, we did not notice the expression of β2, β3, β4 and β5 in D283 cells. (B) Total cell lysates were extracted from non-irradiated and irradiated cells and subjected to western blotting to determine the phosphorylation levels of FAK, Src and Paxillin and Rac-1 in DAOY and D283 cells.
(0.90 MB TIF)

Figure S2 Graphical representation of the western blot data of Figure 4. (A) The densitometry analysis of the western blots of DAOY and D283 cells transiently transfected with full length (FL-) uPAR as per Figure 4A was carried out. The protein intensity was measured and represented graphically (mean from three independent experiment ± S.D; p<0.05). (B) The densitometry analysis of the western blots of DAOY and D283 of Figure 4B where the cells were treated with or without FAK inhibitor, before subjecting to irradiation. Intensity of protein signals were quantified by densitometer analysis and represented graphically. Experiment was carried out in triplicates with a mean ± S.D (p<0.05).
(0.30 MB TIF)

Figure S3 Effect of uPAR siRNA expressing plasmid treatment prior to radiation treatment on uPAR and phosphorylated FAK expression levels in pre-established intracranial tumor. Immunohistochemical analysis was carried out by probing the brain tissue section with uPAR and phospho FAK (Y397) antibodies. After secondary antibody incubation, the protein expression was detected using 3, 3-diaminobenzidine substrate solution. Sections were further counterstained with hematoxylin and visualized under an inverted microscope.
(6.79 MB TIF)

Table S1 The list of primer used in the present study and their 5′-3′ sequence are given.
(0.05 MB DOC)
